RETRACTED

# Effect of Moxibustion Instrument Combined with Intermediate Frequency Electrostatic Therapy on Pain and Joint Function in Elderly Patients with Cold-Dampness Knee Arthritis

**DOI:** 10.1155/2022/2613901

**Published:** 2022-05-05

**Authors:** Leilei Cui, Zhaoliang Bai

**Affiliations:** ^1^The 971st Navy Hospital of the Chinese People's Liberation Army, The First Outpatients, Qingdao, Shandong 266071, China; ^2^Outpatient Department, 971st Hospital, People's Liberation Army Navy, Qingdao, Shandong 266071, China

## Abstract

**Objective:**

To explore the effect of a moxibustion instrument combined with intermediate frequency electrostatic therapy on pain and joint function in elderly patients with cold-dampness arthritis (KOA).

**Method:**

200 patients with cold-dampness KOA treated in our hospital from May 2019 to September 2021 were selected. According to the random number table method, they were divided into the observation group (*n* = 100) and control group (*n* = 100). The observation group was treated with moxibustion combined with medium-frequency treatment, and the control group was treated with medium-frequency treatment. The clinical effects of the two groups were compared. The joint functions of the two groups were evaluated by the visualization scale of the osteoarthritis index (WOMAC index) of McMaster University in Western Ontario. The TCM symptom scores of the two groups were evaluated according to the guiding principles for clinical research of new traditional Chinese medicine. The visual analogue scale (VAS) was used to evaluate the pain degree of the two groups, and the microcirculatory blood perfusion (MBPU) and interleukin-1 were compared between the two groups, *β* (IL-1*β*) and tumor necrosis factor-*α* (TNF-*α*). The levels of matrix metalloproteinase-1 (MMP-1), serum bone morphogenetic protein-2 (BMP-2), cartilage oligomeric matrix protein (COMP), and serum type II collagen C-terminal peptide (CTX-II) were assessed by the comprehensive quality of life questionnaire-74.

**Result:**

The total effective rate of the observation group (92.00%) was higher than that of the control group (76.00%), and the difference was statistically significant (*P* < 0.05) in *β* and TNF-*α*. The levels of MMP-3, BMP-2, comp, and CTX-II and the improvement of quality of life score in the control group were better than those in the control group (*P* < 0.05).

**Conclusion:**

Moxibustion instrument combined with intermediate frequency electrostatic therapy can effectively improve the knee joint function, pain, blood perfusion, inflammatory reaction, and cartilage damage of the elderly patients with cold-dampness-type knee arthritis, and the therapeutic effect is good.

RETRACTED

## 1. Introduction

Osteoarthritis is a common degenerative disease in clinics. Its main clinical manifestations are joint swelling and pain and stiffness which can lead to disability. Osteoarthritis mainly occurs in the knee joint and hip joint, and it is common in middle-aged and elderly patients with a high incidence. According to relevant research, the incidence of the bone joint in the middle-aged and elderly people over 40 years old in China has reached 46.3%, of which 15.6% is knee osteoarthritis (KOA), which can seriously affect the quality of life of patients and bring heavy burden to patients' families and society [1, 2]. At present, anti-inflammatory, analgesic, and intra-articular injection or surgical treatment is mostly used in the clinical treatment of osteoarthritis of the knee joint, with a good short-term curative effect, but the condition is easy to repeat [3, 4]. Besides surgery, the treatment modalities include exercise, knee braces, walking aids, oral NSAIDs, and surgery. Oral NSAIDs are commonly used medicine to alleviate KOA-associated pain. However, long-term use of NSAIDs is often associated with cardiovascular diseases such as myocardial infarction, kidney injury, and gastrointestinal symptoms [5]. Therefore, alternative nonpharmacological interventions to alleviate KOA symptoms are in high demand. KOA belongs to the category of “bone arthralgia” in traditional Chinese medicine. Deficiency of kidney-qi, deficiency of kidney-yang, stagnation of qi and blood stasis, and cold coagulation of meridians can all lead to blockage of meridians, and obstruction will cause pain. For elderly patients, the pathogenesis of KOA is complicated, and there are many cases of mixed cold and heat and mixed deficiency and excess. The physique of the elderly is mostly in the state of liver and kidney deficiency and old age strain, with the loss of qi, blood, and yin and yang. They are vulnerable to exogenous pathogens such as wind, cold, and dampness, which can cause arthralgia of joints and meridians, affect the movement of qi and blood, and eventually lead to cold coagulation and stasis, arthralgia, and cold-dampness KOA [6, 7]. Moxibustion is a traditional Chinese medicine treatment method. Acupuncture can dredge meridians, and moxibustion has the functions of warming qi and blood, strengthening vital energy, and eliminating evil. Warm acupuncture refers to the combination of acupuncture and moxibustion. Traditional warm acupuncture has some shortcomings. It usually burns the skin and causes infection. The moxibustion instrument can completely replace traditional warm acupuncture and avoid scalding patients and can improve the working efficiency of medical staff. It belongs to medium-frequency physiotherapy. The principle of action is that two groups of electrodes cross-act on the affected part of the human body to generate a dynamic bioelectric field and then generate current along the direction of the bone axis to activate chondrocytes, accelerate cell metabolism, promote callus formation, and have a good effect of treating arthralgia. The purpose of this study is to explore the effect of moxibustion instrument combined with intermediate frequency electrostatic therapy on joint pain and joint function of KOA in the elderly with cold-dampness type, which is reported as follows.

RETRACTED

## 2. Materials and Methods

### 2.1. General Information

200 patients with cold-dampness KOA treated in our hospital from May 2019 to September 2021 were randomly divided into observation group and control group, with 100 cases in each group. There were 44 males and 56 females in the observation group, aged 60-85 years. The average age was 72.00 ± 6.00 years; the course of the disease was 1~6 years, with an average of 2.76 ± 1.48 years; there were 37 cases of unilateral disease and 63 cases of bilateral disease; there were 33 cases of X-ray grade I, 43 cases of grade II, and 24 cases of grade III. There were 48 males and 52 females in the control group; the age was 60~93 years, with an average of 70.78 ± 6.16 years; the course of the disease was 1~6 years, with an average of 2.82 ± 1.53 years; there were 43 cases of unilateral disease and 57 cases of bilateral disease; there were 30 cases of X-ray grade I, 37 cases of grade II, and 33 cases of grade III. The general data of the two groups were comparable (*P* > 0.05). There were no significant differences in the joint functions, the TCM symptom scores, and the visual analogue scale between the 2 groups before intervention (*P* > 0.05; Table 1). This study was approved by the hospital ethics committee.

The inclusion criteria are as follows: (1) all met the requirements of bone and joint diagnosis and treatment (2018 edition) [8]. According to the diagnostic criteria of KOA, there was a history of trauma, repeated strain, knee pain, stiffness, aggravation of pain during activity, friction sound, etc., and there was a lip-like hyperplasia at the joint edge in imaging examination. (2) They all meet the diagnostic criteria of cold-dampness obstruction syndrome in the guiding principles for clinical research of new traditional Chinese medicine [9] and the diagnostic criteria of TCM syndrome types: diagnostic and curative effect criteria of TCM diseases [10]. (3) Age ≥ 60 years. (4) TCM syndrome differentiation is a cold-dampness syndrome. The standard of the cold-dampness syndrome is that the joints and muscles are painful and sour, and the joints cannot be flexed and extended. It can involve multiple joints. In the case of cold, the pain will be abundant, in the case of heat, the pain will be slow, the tongue will be light, the fur will be white, and the pulse will float. (5) Immunosuppressants and glucocorticoids were not used, and nonsteroidal anti-inflammatory drugs and cytotoxic drugs were not used 1 day before blood collection. (6) They all volunteered to participate in this study.

RETRACTED

The exclusion criteria are as follows: (1) patients will be excluded if they have nonprimary knee osteoarthritis (secondary knee osteoarthritis, inflammatory, or other rheumatic diseases); (2) patients with autoimmune diseases; (3) patients with severe organ dysfunction such as heart, liver, and kidney; (4) patients with mental illness; (5) patients with internal and external collateral ligament injury of the knee joint; (6) patients with severe bone tumor, osteoporosis, early fracture, and early paraplegia; (7) complicated with severe basic diseases; and (8) patients with bladder dysfunction.

### 2.2. Methods

The control group was treated with medium-frequency static electricity (K8832-T), while the observation group was treated with medium-frequency static electricity combined with the moxibustion instrument (G-6805). In intermediate frequency electrostatic therapy, the intermediate frequency electrostatic therapeutic apparatus is used for the treatment. Before use, the basic principle, performance, and therapeutic effect of the apparatus are informed to the patients, and their consent is obtained. The red and white electrode pads were placed opposite to each other or side by side in the affected part of the knee joint, and the high-voltage electrostatic mode was selected for 15 min/time, twice/day, with 5 days as a course of treatment, and both groups were treated for 2 courses of treatment. The distance between the two electrodes is 4 cm~9 cm, and the selected intensity is 0.1. The distance between the two electrodes is 9 cm~13 cm, and the selected intensity is 0.2. The distance between the two electrodes is greater than 13 cm, and the selected intensity is 0.3. The therapeutic apparatus is operated by a special person. If the patient feels that the strength of the electrode sheet is unequal during the operation, he should stop and find out the reason to decide whether to continue the treatment. During the treatment, pay attention to observe the patient's condition and ask if the patient has tension and severe pain in the treatment area. In moxibustion therapy, the patient takes a sitting position, the knee joint flexes at 90 degrees, Xuehai and Liang Qiu are selected for vertical needling, the needling depth is 1~1.5 inches, the inner and outer knee eyes use 3-inch millineedles, the needle tip pierces 2~2.5 inches into the center of the knee joint, then twists and turns after getting angry, and the deep part of the knee joint feels sore and swollen. Leave the needle, place the moxibustion head of the moxibustion instrument, open a small hole in the center of four round moxa bags with triangular needles, pass the moxa bags through the needle handles through this hole, put them on the moxa pads, cross-fix them with 2 strips of 1 cm × 20 cm long adhesive tapes, set the temperature of each moxibustion head of the moxibustion instrument, keep it for 30 minutes, twist the needle handles twice in the middle, and then remove the adhesive tapes, moxibustion heads, and moxa pads. The treatment frequency was 3 times/week, a total of 10 times.

RETRACTED

### 2.3. Observation Index

The observation index includes the following: (1) clinical efficacy. (2) Joint function was evaluated by the Western Ontario Macmaster University osteoarthritis index (WOMAC Index) [11], which included pain score (5 items, 0-20 points), joint stiffness score (2 items, 0~8 points), and daily activity score (17 items, 0~68 points). The score from inaction to the extreme is (0~4 points) with a total score of 0~96 points before and after treatment. (3) TCM symptom scores were evaluated by the “Guiding Principles of Clinical Research on New Drugs of Traditional Chinese Medicine” before and after treatment [9]. The main symptoms were severe joint pain, which aggravated in cold and decreased in temperature. The scores were 0, 2, 4, and 6 from no, light, medium, and heavy. The second symptom is waist and waist pain. No, light, medium, and heavy symptoms are scored according to 0, 1, 2, and 3. The higher the score, the more severe the symptoms of patients. (4) The degree of pain in the two groups was evaluated by the visual analogue scale (VAS) before and after treatment [12]. The total score was 0~10 points, mild pain (1~3 points), moderate pain (4~6 points), and severe pain (7~10 points). The higher the score, the more severe the pain symptoms were. (5) In microcirculation blood flow perfusion (MBPU), set the room temperature to 26~28°C, and rest for 10 minutes before the test to adapt to the indoor environment. The subjects took an upright position, the height of the seat was adjusted to make the affected side bend their hips and knees by 90 degrees, the blood flow perfusion was detected at 0.5 cm next to the nasal acupoint with the laser Doppler blood flow meter, the time was set constant to 0.2 s, and the blood flow perfusion was detected with the Temp Unit temperature control unit. (6) Blood samples were collected before and after treatment. Inflammatory factors are as follows: Take 5 ml of fasting venous blood from two groups in the morning, centrifuge at 3000 r/min and 8 cm radius for 10 min, and take the upper serum to be tested, and the levels of interleukin- (IL-) 1*β*, tumor necrosis factor-*ι* (TNF-*ι*) and mechanism metalloproteinase-3(MMP-3) are determined by the enzyme-linked immunosorbent assay. (7) Blood samples were collected before and after treatment. The levels of serum bone morphogenetic protein 2 (BMP-2), cartilage oligomeric matrix protein (COMP), and serum C-terminal peptide of type II collagen (CTX-II) were taken from the above serum, and the levels of BMP-2, COMP, and CTX-II were determined by the enzyme-linked immunosorbent assay. (8) The quality of life is evaluated by the comprehensive quality of life assessment questionnaire-74 [13], which includes four dimensions, four factors in each dimension, and a total of 16 factors (64 items). The highest score of each factor is 20 points, and the highest score of each dimension is 80 points. The higher the score, the better the quality of life. (9) Efficacy evaluation criteria are as follows: The grading and quantitative scores of pain, joint stiffness, daily activity symptoms, and signs of the two groups were evaluated according to the guiding principles for clinical research of new traditional Chinese medicine [9]. The improvement percentage of main symptoms and signs was calculated as (%) = (pretreatment value − posttreatment value)/pretreatment value × 100%. In clinical recovery, the scores of pain, swelling, and other symptoms are reduced by more than 95%, and the patient's joints can move positively. The remarkable effect is as follows: pain, swelling, and other symptoms will reduce the score by about 70%~95%, and the joint activity is not limited. Effective results are as follows: the scores of symptoms and signs such as pain and swelling are reduced by 30%~69%, and the patient's joint activity is improved. Ineffective results are as follows: the scores of symptoms and signs such as pain and swelling were reduced by <30%. Total effective = clinically cured + markedly effective + effective. (10) The occurrence of adverse reactions was recorded, including burns, bleeding, infection, headache, nausea, vomiting, and dizziness.

RETRACTED

### 2.4. Statistical Method

The SPSS 20.0 statistical software was used to analyze and process the data. The measurement data were expressed as *x* ± *s*. An independent sample *t*-test was performed for the comparison between groups. Paired *t*-test was used for the comparison before and after treatment. The counting data were expressed as frequency and constituent ratio, and the *χ*^2^ test was performed. *P* < 0.05 indicates that the difference was statistically significant.

## 3. Result

### 3.1. Comparison of the Clinical Efficacy between the Two Groups

The total efficiency (92.00%) was higher than the control group (76.00%), and the difference was statistically significant (*P* < 0.05; Table 2).

### 3.2. Comparison of the WOMAC Scores between the Two Groups

The SPSS 20.0 statistical software was used to analyze and process the data. The measurement data were expressed as *x* ± *s*. An independent sample *t*-test was performed for the comparison between groups. Paired *t*-test was used for the comparison before and after treatment. The counting data were expressed as frequency and constituent ratio, and the *χ*^2^ test was performed. *P* < 0.05 indicates that the difference was statistically significant (Table 3).

### 3.3. Comparison of TCM Syndrome Points between the Two Groups

Before treatment, there was no significant difference in knee joint pain and waist pain scores between the two groups (*P* > 0.05). After treatment, the scores of knee joint pain and waist pain in both groups decreased, and the observation group was lower than the control group, with statistical significance (*P* < 0.05; see Table 4).

### 3.4. Comparison of Pain and Blood Flow Perfusion between the Two Groups

Before treatment, the VAS score and MBPU value did not differ (*P* > 0.05), the VAS score and MBPU value decreased, and the observed group was significant (*P* < 0.05; see Table 5).

### 3.5. Comparison of the Inflammatory Factor Levels between the Two Groups

Before treatment, there was no difference in serum IL-1, TNF, and MMP-1 levels (*P* > 0.05), serum IL-1, TNF, and MMP-1 decreased, and the observed group was lower than the control group, statistically significant (*P* < 0.05; see Table 6).

### 3.6. Comparison of BMP-2, COMP, and CTX-II Levels between the Two Groups

Before treatment, there was no difference in serum BMP and CTX-II levels (*P* > 0.05); after treatment, the serum BMP-2, COMP, and CTX-II decreased, and the observed groups were significantly different (*P* < 0.05; see Table 7).

### 3.7. Comparison of Quality of Life between the Two Groups

Before treatment, there was no significant difference in scores of quality of life between the two groups (*P* > 0.05). After treatment, the scores of all dimensions of quality of life in the two groups increased, and the observation group was higher than the control group, with statistical significance (*P* < 0.05; see Table 8).

### 3.8. Untoward Effect

No serious adverse reactions occurred in both groups.

RETRACTED

## 4. Discussion

Knee arthritis belongs to “bone arthralgia” in traditional Chinese medicine. There are many causes of this disease. Patients' lack of healthy qi, weak external health, or congenital deficiency can all lead to wind-cold-damp-heat taking advantage of it, which leads to poor qi and blood movement, obstruction of meridians, and obstruction of muscles, joints, and meridians of patients, which leads to pain. The external symptoms are swelling of the knee joint, pain and stiffness of limbs, and inability to move flexibly. Therefore, the method of eliminating evil, dispelling wind, dispelling cold, and dredging meridians should be adopted to treat this disease. In this study, a moxibustion instrument combined with medium-frequency electrotherapy is used. Moxibustion therapy is one of the traditional Chinese medicine treatment methods, which has the functions of hyperthermia, phototherapy, drug stimulation, and acupoint stimulation. The warmth of moxa fire is transmitted to the skin through the needle body, and it has the functions of activating collaterals, dispelling cold, and relieving pain. Moxibustion at Xuehai point can promote blood circulation and dispel wind, and moxibustion at Liangqiu point can tonify qi and blood. Modern pharmacological research shows that the light energy and heat energy generated by burning mugwort leaves can effectively improve the vascular permeability, reduce the blood concentration and aggregation, reduce the inflammatory stimulation, accelerate the removal of local pathological wastes, and finally effectively improve the pain of knee arthritis [14, 15]. Medium-frequency electrotherapy is a common clinical physiotherapy scheme, which can accelerate the release of endogenous morphine in the central nervous system, promote cell metabolism and the formation of intracellular cyclic adenosine monophosphate, have anti-infection and analgesic effects, effectively improve capillary permeability, relieve patients' pain, enhance muscle strength, and promote the recovery of patients' knee joint function [16]. This is a randomized, assessor-blinded clinical trial to explore the effect of the moxibustion instrument combined with intermediate frequency electrostatic therapy on pain and joint function in elderly patients with cold-dampness arthritis.

In this study, the total effective rate of the observation group (92.00%) was higher than that of the control group (76.00%). After treatment, the improvement degree of WOMAC score, TCM syndrome score, and VAS score in the observation group is better than that in the control group, which indicates that moxibustion instrument combined with intermediate frequency electrostatic therapy can effectively improve the joint function, clinical symptoms, and pain of patients. The moxibustion instrument can improve blood vessel permeability, activate collaterals, relieve pain through thermotherapy, phototherapy, drug stimulation, and acupoint stimulation, and finally improve knee joint function [17]. Intermediate frequency electrostatic therapy can promote cell metabolism, improve pain, enhance muscle strength, and improve joint function. Both of them play a multitarget therapeutic role, so the improvement of knee joint function, clinical symptoms, and pain in the observation group is better than that in the control group. Previous studies have shown that the moxibustion instrument combined with physical therapy can also improve the knee joint function of patients more effectively, and the results of this study are consistent with that [18]. Microcirculation is the basic structure of the circulatory system, which is closely related to the material exchange between tissues, and can directly affect the development and outcome of arthritis. MBPU represents the product of the number of blood cells passing through monitoring points and the moving speed per unit of time. In this study, after treatment, the MBPU value of the observation group was significantly lower than that of the control group, indicating that the improvement of blood perfusion in the microcirculation of the knee joint was better than that of the control group, and its mechanism might be related to the improvement of local temperature, microcirculation, and vascular permeability by moxibustion instrument.

RETRACTED

Previous studies have shown that the occurrence and development of knee arthritis are closely related to inflammatory factors, and the levels of serum IL-1*β*, TNF-*α*, and MMP-1 in patients with knee arthritis are significantly increased [19–21]. IL-1*β* is an inflammatory cytokine, which can participate in many pathological processes such as tissue destruction and edema, and can stimulate synovial inflammation. TNF-*α* is involved in various inflammatory reactions, closely related to joint destruction, rheumatoid arthritis injury degree, and inflammation, and involved in the onset of senile knee arthritis and cartilage injury process. MMP-1 is a degradation enzyme of articular cartilage and plays an important role in the process of cartilage degeneration. The pain degree of KOA is closely related to the severity of joint inflammation which can be determined or reflected by the levels of inflammation-related factors. Therefore, understanding the state of cytokines in the synovial fluid before and after treatment is an approach to assess the efficacy of our treatment [22]. In this study, after treatment, the improvement degree of serum IL-1*β*, TNF-*α*, and MMP-1 levels in the observation group is greater than that in the control group, which indicates that moxibustion instrument combined with intermediate frequency can effectively improve the inflammatory state of patients, which may be related to the light and heat energy generated by moxibustion instrument.

RETRACTED

BMP, COMP, and CTX-II are the markers of cartilage metabolism. BMP-2 has been suggested as a tool for cartilage repair and a stimulant of chondrogenesis. BMP-2 is rarely present in healthy cartilage, whereas it is highly expressed in osteoarthritis. BMP-2 can induce chondrogenesis in human mesenchymal stem cells in vitro [23]. COMP is an extracellular glycoprotein, whose level can damage the collagen-fiber network of articular cartilage and aggravate cartilage damage. CTX-II is a small molecule peptide produced by the stimulation of type II collagen by protease, and its level reflects the degradation ability of type II collagen, which is involved in the degeneration of articular cartilage and the formation of KOA [24]. The levels of serum BMP-2, COMP, and CTX-II in patients with osteoarthritis of the knee can be significantly increased [25, 26]. By regulating the synthesis and activation of cytokines, the damage of articular cartilage can be alleviated, and its stability can be improved. In this study, after treatment, the improvement of serum BMP-2, COMP, and CTX-II levels in the observation group was greater than that in the control group. It shows that the moxibustion instrument combined with intermediate frequency can more effectively regulate the synthesis and activation of cytokines in patients with knee arthritis, which may be related to the stimulation, light, and heat effects of the moxibustion instrument on acupoints, and its specific mechanism needs to be further explored. Compared with the quality of life of the two groups, after treatment, the improvement degree of the quality of life of the observation group was significantly better than that of the control group, the knee joint function of the patients in the observation group recovered better, and the pain improvement was also better than that of the control group, so the quality of life was significantly improved. This study underwent 10 times of treatment because of the limited time. We had scheduled a follow-up visit with our patient in a few months.

To sum up, the moxibustion instrument combined with intermediate frequency can effectively improve the knee joint function and clinical symptoms of elderly patients with cold-dampness knee osteoarthritis, effectively relieve their pain, improve their blood flow perfusion, and relieve their inflammatory reaction, which has clinical application value.

RETRACTED

## Figures and Tables

**Table 1:** Comparison of the general information between the two groups.

Groups	Observation group (*n* = 100)	Control group (*n* = 100)	*P* value
Gender (male/female) (*n*)	44/56	48/52	0.911
Age (years old)	72.00 ± 6.00	70.78 ± 6.16	0.736
Course (years)	2.76 ± 1.48	2.82 ± 1.53	0.750
Unilateral disease/bilateral disease (*n*)	37/63	43/57	0.059
X-ray grade (I/II/III)	33/43/34	30/37/33	0.176

**Table 2:** Comparison of the clinical efficacy between the two groups (case (%)).

Groups	Clinical recovery	Excellence	Effective	Invalid	Total effective
Observation group (*n* = 100)	33 (33.00)	45 (45.00)	14 (14.00)	8 (8.00)	92 (92.00)
Control group (*n* = 100)	11 (11.00)	33 (33.00)	32 (32.00)	24 (24.00)	76 (76.00)
*χ* ^2^ value					9.524
*P* value					0.002

**Table 3:** Comparison of WOMAC scores between two groups (*x* ± *s*, points).

Groups	Pain score		Joint stiffness score		Daily activity score		Aggregate score	
	Prior treatment	Posttreatment	Prior treatment	Posttreatment	Prior treatment	Posttreatment	Prior treatment	Posttreatment
Observation group (*n* = 100)	10.79 + 1.42	4.29 + 1.47^a^	6.05 + 1.08	1.38 + 0.79^a^	51.02 + 5.47	22.26 + 2.13^a^	67.89 + 5.96	27.93 + 2.60^a^
Control group (*n* = 100)	10.97 + 1.32	6.78 + 1.61^a^	5.91 + 1.02	2.64 + 1.42^a^	50.28 + 5.06	30.43 + 3.51^a^	67.16 + 4.94	39.85 + 4.17^a^
*T* value	0.927	11.455	0.946	7.766	0.993	19.894	0.904	24.234
*P* value	0.355	<0.001	0.345	<0.001	0.322	<0.001	0.367	<0.001

Note: compared with the same group before treatment, ^a^*P* < 0.05.

**Table 4:** Comparison of TCM credits (*x* ± *s*, points).

Groups	Knee pain		Heavy pain in the waist	
	Prior treatment	Posttreatment	Prior treatment	Posttreatment
Observation group (*n* = 100)	3.74 + 0.79	1.20 + 0.98^a^	1.73 + 0.53	0.48 + 0.50^a^
Control group (*n* = 100)	3.78 + 0.69	1.76 + 0.65^a^	1.82 + 0.66	0.74 + 0.58^a^
*T* value	0.382	4.739	1.067	3.391
*P* value	0.703	<0.001	0.287	0.001

Note: compared with the same group before treatment, ^a^*P* < 0.05.

**Table 5:** Comparison of pain and blood flow perfusion in the two groups (*x* ± *s*).

Groups	VAS score (score)		MBPU	
	Prior treatment	Posttreatment	Prior treatment	Posttreatment
Observation group (*n* = 100)	6.33 + 1.40	1.77 + 0.84^a^	12.48 + 1.26	7.42 + 1.65^a^
Control group (*n* = 100)	6.39 + 1.32	3.68 + 1.29^a^	12.24 + 1.11	8.71 + 1.44^a^
*T* value	0.311	12.438	1.421	5.911
*P* value	0.756	<0.001	0.157	<0.001

Note: compared with the same group before treatment, ^a^*P* < 0.05.

**Table 6:** Comparison of inflammatory levels between the two groups (*x* ± *s*).

Groups	IL-1*β* (ng/l)		TNF-*α* (*μ*g/l)		MMP-1 (ng/l)	
	Prior treatment	Posttreatment	Prior treatment	Posttreatment	Prior treatment	Posttreatment
Observation group (*n* = 100)	5.36 + 1.19	1.08 + 0.23^a^	8.32 + 2.15	2.22 + 0.91^a^	359.33 + 35.43	89.21 + 8.04^a^
Control group (*n* = 100)	5.50 + 0.91	3.49 + 0.57^a^	8.49 + 2.18	4.06 + 1.15^a^	361.65 + 36.73	168.31 + 16.34^a^
*T* value	0.952	39.494	0.553	12.620	0.455	43.440
*P* value	0.342	<0.001	0.581	<0.001	0.650	<0.001

Note: compared with the same group before treatment, ^a^*P* < 0.05.

RETRACTED

**Table 7:** Comparison of BMP-2, COMP, and CTX-II levels between the two groups (*x* ± *s*).

Groups	BMP-2 (ng/ml)		COMP (U/l)		CTX-II (*μ*g/l)	
	Prior treatment	Posttreatment	Prior treatment	Posttreatment	Prior treatment	Posttreatment
Observation group (*n* = 100)	1.86 + 0.45	0.79 + 0.17^a^	13.39 + 3.38	8.17 + 2.28^a^	581.63 + 58.17	440.54 + 37.35^a^
Control group (*n* = 100)	1.88 + 0.31	1.42 + 0.30^a^	13.95 + 3.29	9.78 + 2.74^a^	579.66 + 47.53	492.66 + 50.00^a^
*T* value	0.233	18.016	1.205	4.528	0.262	8.351
*P* value	0.816	<0.001	0.230	<0.001	0.794	<0.001

Note: compared with the same group before treatment, ^a^*P* < 0.05.

**Table 8:** Comparison of quality of life between two groups (*x* ± *s*, score).

Groups	Somatic function		Mental function		Social function		Material life function	
	Prior treatment	Posttreatment	Prior treatment	Posttreatment	Prior treatment	Posttreatment	Prior treatment	Posttreatment
Observation group (*n* = 100)	45.82 + 3.12	71.60 + 6.35^a^	46.22 + 3.67	73.38 + 6.33^a^	46.01 + 4.02	67.90 + 6.57^a^	50.73 + 6.08	71.01 + 8.52^a^
Control group (*n* = 100)	45.46 + 4.40	59.31 + 4.71^a^	47.04 + 4.46	58.08 + 4.61^a^	46.34 + 4.41	58.86 + 4.82^a^	49.60 + 6.22	62.00 + 6.04^a^
*T* value	0.668	15.541	1.419	19.525	0.554	11.091	1.299	8.628
*P* value	0.505	<0.001	0.157	<0.001	0.580	<0.001	0.196	<0.001

Note: compared with the same group before treatment, ^a^*P* < 0.05.

## Data Availability

The labeled dataset used to support the findings of this study is available from the corresponding author upon request.
